# HIV and COVID-19 Coinfection: A Synergism That Results in More Severe Forms of Reactive Arthritis

**DOI:** 10.7759/cureus.19396

**Published:** 2021-11-09

**Authors:** Juan Camilo Santacruz, Marta Juliana Mantilla, Sandra Pulido, Angelo Arzuaga, Juan Manuel Bello, John Londono

**Affiliations:** 1 Spondyloarthropathies Research Group, Universidad de La Sabana, Chía, COL; 2 Rheumatology, Universidad Militar Nueva Granada, Bogotá, COL

**Keywords:** reactive arthritis, polyarticular compromise, covid 19, hiv, immune system

## Abstract

Reactive arthritis is defined as arthritis that arises after infection, where pathogens cannot grow in the affected joints. Although the human immunodeficiency virus and severe acute respiratory syndrome coronavirus 2 are not among the most commonly implicated pathogens, there is growing evidence that they have major implications in the genesis of reactive arthritis. However, there are no described cases of coinfection of both entities that cause reactive arthritis at the same time, and the alterations involved in the immune system that could cause the change of certain clinical characteristics to more severe forms of the disease are unknown. The following describes the case of a male patient in his third decade of life who has an unusual and severe presentation of reactive arthritis associated with coinfection by COVID-19 and the human immunodeficiency virus.

## Introduction

The term "reactive arthritis" (ReA) was introduced in 1969 as an arthritis that appeared shortly after or during infection without achieving the identification of the microorganism in the joint tissue [1]. The original definition did not specify the pathogens that were accepted as causes of ReA and, in 1999, a panel of experts determined a specific list of gastrointestinal and urogenital pathogens that could be considered as possible causative agents [2]. Additionally, certain bacterial or viral respiratory infections (particularly COVID-19) have been associated with certain cases of ReA [3]. The human immunodeficiency virus (HIV) has also been associated as the causative agent of several joint syndromes, the most frequent being seronegative spondyloarthritis, rheumatoid arthritis, and joint pain syndrome [4]. However, some authors have considered that the cause of ReA in these cases is more related to exposure to other infections than to HIV per se [5]. Despite this, there is growing evidence today increasingly supporting the role of HIV as a possible cause of ReA. At present, it is unknown how COVID-19 infection can potentiate the immunosuppressive state caused by HIV, leading to more severe and atypical presentation of ReA along with the additional implication of limiting immunosuppressive treatment due to the inherent risk of potentially life-threatening infection.

## Case presentation

A 27-year-old male patient was admitted to a high-complexity institution due to a five-day clinical picture consisting of additive, symmetrical polyarticular pain, located in the wrists, knees, and left shoulder without other associated symptoms. The joint pain was continuous, permanent, and of great intensity that caused limitation of movement, mainly in the hands. In the systems review, no urinary or gastrointestinal symptoms were documented before the onset of joint symptoms. As the only relevant antecedent, he referred mild respiratory infection by severe acute respiratory syndrome coronavirus 2 (SARS-CoV-2) confirmed by reverse transcription-polymerase chain reaction the month before hospitalization. The initial clinical examination confirmed the presence of bilateral carpal synovitis, left suprapatellar synovitis, and synovitis of the sternoclavicular joints (Figures 1, 2, 3).

**Figure 1:** Left carpal synovitis

 

**Figure 2:** Left suprapatellar synovitis

**Figure 3:** Sternoclavicular joint synovitis

Magnetic resonance imaging of the different compromised anatomical compartments was performed, presenting as additional findings the presence of bursitis of the lateral collateral ligament of the left lower limb and a peritendinous inflammatory process of the triangular fibrocartilage in the right wrist. Mild lymphopenia associated with a marked elevation of acute-phase reactants was documented in laboratory studies. Differential diagnoses of infectious etiology were sought, including a positive fourth-generation HIV enzyme-linked immunosorbent assay with a subsequent CD4 count of 98 cells/mm^3^ and a viral load of 459,000 copies/mL. Treatment with prednisolone at a dose of 1 mg/kg and sulfasalazine (1 g per day) was initiated and no significant improvement in joint symptoms was noted despite sequential changes from disease-modifying antirheumatic drugs (DMARDs) such as methotrexate and leflunomide. Subsequently, the patient achieved a complete joint response when antiretroviral therapy (abacavir, dolutegravir/lamivudine) was initiated, thereby achieving a response to therapy resulting in gradual reduction of glucocorticoid doses and tapering to maintenance therapy solely with sulfasalazine. The description of the most representative laboratory studies upon admission and during hospitalization is shown in Table 1.

**Table 1:** Laboratory parameters at admission and during hospitalization ANAS: antinuclear antibodies; Anti-HBc Ab: hepatitis B core total antibodies; CRP: C-reactive protein; ENAS: extractable nuclear antigens; ESR: erythrocyte sedimentation rate; HBsAg: hepatitis B surface antigen; HIV: human immunodeficiency virus; HLA: human leukocyte antigen; VDRL: Venereal Disease Research Laboratory

Laboratory studies	Upon admission	Hospitalization
Hemoglobin (g/dL)	12.6	12.5
Total leukocyte count (/µL)	7920	8006
Total lymphocyte count (/µL)	960	1200
Total platelet count (/µL)	176,000	213,000
Creatinine (mg/dL)	0.81	0.83
Ureic nitrogen (mg/dL)	11.9	8.3
CRP (mg/dL)	15.9	27
ESR (mm/h)	68	88
Ferritin (ng/mL)	829	-
HBSAg	Non-reactive	-
Anti-HBc Ab	Non-reactive	-
VDRL	Non-reactive	-
HIV	Reactive	-
CD4 + (cells/mm^3^)	98	-
HIV viral load (copies/mL)	459,000	-
ANAS (titers)	Non-reactive	-
ENAS (U/mL)	Non-reactive	-
HLA - B27	Negative	-
Rheumatoid factor (U/mL)	Negative	-
Anti-citrulline antibodies (U)	Negative	-
Uroanalysis	Negative for infection	Negative for infection

## Discussion

In the cases of ReA associated with HIV, the most characteristic presentation is an asymmetric oligoarthritis that more frequently involves the lower extremities associated with enthesitis. Extra-articular cutaneous manifestations such as blennorrhagic keratoderma and circinate balanitis are also common. Additionally, these patients can present extensive psoriasiform lesions that can even be confused with psoriatic arthritis [6]. Paradoxically, urethritis occurs with a similar frequency to patients with ReA without HIV. Axial involvement and uveitis are very rare forms of presentation. The distribution of HLA-B27 positivity is very heterogeneous, with a high frequency in Caucasians (80-90%) with almost absolute negativity in African patients [7]. A lower frequency of involvement of the hand and wrist joints and multidigital dactylitis has also been described [8]. It is noteworthy that joint symptoms can manifest at any time during the course of the disease, but appear to be more frequent in the later stages of the infection [9]. The clinical course can vary from a mild joint involvement with a good response to the use of non-steroidal anti-inflammatory drugs, to a severe clinical picture, characterized by periostitis and multiple radiographic erosions [10]. Within the immunopathogenesis of ReA and its association with HIV, several theories have been proposed. The first one is that the acquired immunodeficiency syndrome (AIDS) would predispose the individual to bacterial, viral, and parasitic joint infections caused by arthritic microorganisms, which would favor the appearance of ReA. Another possibility would be that the immune dysfunction caused by AIDS would lead to an increase in the number of CD8+ T cells, with a reduction in CD4+ T cells, implicating a modification of immune regulation, with the possible induction of ReA [11]. In cases with HIV and COVID-19 coinfection, additional alterations in the immune system have also been described, such as a decrease in regulatory T cells that contribute to the formation of dysfunctional T cells [12]. It has also been suggested that intestinal CD4+ T cells with mucosal protective T helper 17 functions are rapidly depleted leading to intestinal barrier dysfunction, favoring bacterial translocation and persistent immune activation [13]. It is noteworthy that both HIV-1 and SARS-CoV-2 infection share the loss of CD4+ T cells as a result of the disease-causing immunodeficiency. It has been suggested that both entities can cause direct attacks on CD4+ T cells, perpetuate immune activation, and redistribute CD4+ cells to lymph nodes and the intestine, reducing their concentration in peripheral blood. Additionally, lymphopenia is a hallmark of severe COVID-19 patients and is associated with unfavorable clinical outcomes. Importantly, CD4+ T helper cells are vital in mediating humoral immunity by stimulating B cells to produce antibodies to these viruses. On the other hand, CD8+ T cells are responsible for the elimination of infected cells through the production of perforin and granzyme, being essential for viral control by the secretion of cytokines [14]. The loss of CD4+ T cells in both entities is demonstrated by the increase in biomarkers such as CD38, HLA-DR, and programmed death 1 (PD-1) that are expressed in activated T cells, contributing to their depletion [15]. Depleted virus-specific CD4+ T cells express PD-1 at high levels that correlate with disease progression, higher viral loads, and reduced T cell counts [16]. Regarding the treatment of ReA associated with HIV, it continues to be a controversial issue due to the possible exacerbation of viral infection due to the use of immunosuppressive drugs. However, if the patient does not respond to conventional symptomatic treatment, glucocorticoids and DMARDs should be considered, especially in refractory and persistent cases. Hydroxychloroquine is considered effective and safe among DMARDs, along with possible antiretroviral properties demonstrated in vitro. Sulfasalazine and cyclosporine are considered safe and effective, but experience with the latter is limited [17]. Methotrexate (at doses of 7.5 mg to 15 mg weekly) may also be a treatment option in HIV-infected patients, including those with AIDS, provided that antiretroviral therapy and chemoprophylaxis for *Pneumocystis jirovecii* infection are ensured [18]. The use of anti-tumor necrosis factor (TNF) has been proposed as a viable alternative for patients with HIV infection, without AIDS, who present with ReA refractory to other conventional DMARDs, also insisting on concomitant antiretroviral treatment. Data on the safety of immunomodulatory drugs in people living with HIV are limited. In a study using anti-TNF, antimetabolites, and checkpoint inhibitors, in which 95% of patients received joint antiretroviral therapy, there was a change in viral load (from undetectable to detectable) in the first year of treatment in 41.2%. Additionally, 11.8% of the patients presented an additional severe infection not directly associated with the drug, even with a median CD4+ T cell count of 609 cells/μL. Given these findings, careful monitoring is required to detect signs of virologic relapse and incident infections [19]. Highly effective antiretroviral therapies (HAARTs) have managed to increase the lymphocyte count, improve survival, have changes in the profile of immune responses, and direct cellular metabolic changes, which is why their early initiation is of vital importance [20].

## Conclusions

ReA among patients with HIV and COVID-19 causes important alterations in the innate and adaptive immune system, particularly due to the dysregulation and depletion of T cells, favoring higher levels of immunosuppression. This favors the increase of pro-inflammatory cytokines that can cause a change in the clinical expression of the disease, leading to more serious forms of presentation such as polyarticular involvement. This may also be reflected in the persistent elevation of acute-phase reactants and poor response to DMARDs and glucocorticoids. No studies have been conducted to evaluate the clinical response rates to the use of anti-TNF in patients with AIDS and CD4+ less than 200 cells/mm^3^; however, there is a substantial risk of virological relapse and incident infections even with CD4+ cell counts greater than 200 cells/mm^3^. Concerning the joint response, the risk and benefit of this treatment must be evaluated. HAART therapy is essential to attenuate these alterations in the immune system, achieve early clinical improvement, and be able to have better responses to conventional and biological DMARDs.
